RETRACTED

# Acute Toxicity and Gastroprotection Studies with a Newly Synthesized Steroid

**DOI:** 10.1371/journal.pone.0059296

**Published:** 2013-03-13

**Authors:** Kamal A. Ketuly, A. Hamid A. Hadi, Shahram Golbabapour, Maryam Hajrezaie, Pouya Hassandarvish, Hapipah Mohd Ali, Nazia Abdul Majid, Mahmood A. Abdulla

**Affiliations:** 1 Department of Chemistry, Faculty of Science, University of Malaya, Kuala Lumpur, Malaysia; 2 Department of Molecular Medicine, Faculty of Medicine, University of Malaya, Kuala Lumpur, Malaysia; 3 Institute of Biological Sciences, Faculty of Science, University of Malaya, Kuala Lumpur, Malaysia; University of California, Los Angeles, United States of America

## Abstract

**Background:**

Synthetic steroids, such as 9α-bromobeclomethasonedipropionate, have shown gastroprotective activity. For example, the potent glucocorticoid steroid, beclomethasone dipropionate, has been used for treatment of bowel ulcerations. The purpose of the present study was to evaluate the effect of a synthetic steroid, (20*S*)-22-acetoxymethyl-6β-methoxy-3α,5-dihydro-3′H-cyclopropa[3α,5]-5α-pregnane (AMDCP), on ethanol-induced gastric mucosa injuries in rats.

**Methodology/Principal Finding:**

Rats were divided into 8 groups. The negative control and ethanol control groups were administered Tween 20 (10%v/v) orally. The reference control group, 20 mg/kg omeprazole (10% Tween 20, 5 mL/kg), was administrated orally. The experimental groups received 1, 5, 10, 15 or 20 mg/kg of the AMDCP compound (10% Tween 20, 5 mL/kg). After 60 min, Tween 20 and absolute ethanol was given orally (5 mL/kg) to the negative control group and to the rest of the groups, and the rats were sacrificed an hour later. The acidity of gastric content, gastric wall mucus and areas of mucosal lesions were assessed. In addition, histology and immunohistochemistry of the gastric wall were assessed. Prostaglandin E2 (PGE_2_) and malondialdehyde (MDA) content were also measured. The ethanol control group exhibited severe mucosal lesion compared with the experimental groups with fewer mucosal lesions along with a reduction of edema and leukocyte infiltration. Immunohistochemical staining of Hsp70 and Bax proteins showed over-expression and under-expression, respectively, in the experimental groups. The experimental groups also exhibited high levels of PGE_2_ as well as a reduced amount of MDA. AMDCP decreased the acidity and lipid peroxidation and increased the levels of antioxidant enzymes.

**Conclusion/Significance:**

The current investigation evaluated the gastroprotective effects of AMDCP on ethanol-induced gastric mucosal lesions in rats. This study also suggests that AMDCP might be useful as a gastroprotective agent.

RETRACTED

## Introduction

Peptic ulcers are a common disorder that may occur throughout the entire gastrointestinal tract but mainly occur in the stomach and the proximal duodenum [1]. The gastric mucosal membrane is continuously exposed to potentially harmful agents, such as HCl, pepsin, bile acids, food seasonings, bacterial products and drugs. These agents are involved in the pathogenesis of gastric injury by promoting an increase in the secretion of gastric acid and pepsin and a decrease in gastric blood flow, suppressing the output of endogenous prostaglandins, inhibiting cellular proliferation and growth of the gastric mucosa and altering gastric motility [2]. The basic pathophysiology of gastric ulcers and mucosal lesions results from an imbalance of multiple endogenous aggressive factor(s), such as hydrochloric acid, pepsin, refluxed bile, leukotrienes and reactive oxygen species (ROS) and protective factors, which include a functional mucus-bicarbonate barrier, surface active phospholipids, prostaglandins (PG), mucosal blood flow, cell renewal and migration, non-enzymatic and enzymatic antioxidants and some growth factors [3], [4]. Heat shock proteins, generated by gastric epithelial cells such as Hsp70 are critical macromolecule chaperones [5] which associate in maintaining of physiology of gastric tissue in response to stress, such as oxidative stress through protecting protein against denaturation [6], [7]. Under stress imbalance between anti-apoptotic protein, such as Bcl2 family, and pre-apoptotic protein (Bax) cause gastric ulcer [8]. Several studies evaluated the expression of Hsp70 and Bax to evaluate gastric mucosa protection and damage respectively [9]–[11]. In spite of the multi-faceted pathogenesis of peptic ulcers and mucosal lesions, gastric acid secretion is still recognized as a central component of this disease. Therefore, the main therapeutic goal is to control acid secretion using antacids, H2 receptor blockers (ranitidine and famotidine) or proton pump inhibitors (omeprazole and lansoprazole) [12]. However, current gastric ulcer therapies show limited efficacy against gastric mucosal lesions/ulceration and are often associated with several side effects [4]. In this study, the synthetic steroid acetoxymethyl-6β-methoxy-3α,5-dihydro-3′H-cyclopropa[3α,5]-5α-pregnane (AMDCP) was tested to evaluate its ability to prevent mucosal lesions. Other synthetic steroids, such as 9α-bromobeclomethasone dipropionate, have shown gastroprotective properties at larger dosages [13] than AMDCP. The potent glucocorticoid steroid, beclomethasone dipropionate, has been used for the treatment of bowel ulcerations [14]. However, there is no data in the literature on the gastroprotective activities associated with AMDCP. Hence, the current study was undertaken to evaluate the gastroprotective effects of AMDCP on ethanol-induced gastric mucosal lesions in rats and the effect of ethanol and AMDCP treatment on Hsp70 and Bax proteins in immunohistochemical staining. In addition, the antioxidant status of gastric tissue homogenate was assessed by determining the levels of malondialdehyde (MDA) and Prostaglandin E_2_ (PGE_2_).

RETRACTED

## Materials and Methods

### Omeprazole

In this study, omeprazole (obtained from the University of Malaya Medical Centre (UMMC) Pharmacy) was used as a control for anti-ulcer medicine. The medicine was dissolved in (10% Tween 20, 5 mL/kg) and administered orally to the rats in a single dose of 20 mg/kg body weight (5 mL/kg) according to the recommendations of Mahmood *et al.* [15].

### Synthesis of (20S)-22-Acetoxymethyl-6β-methoxy-3α,5-dihydro-3′H-cyclopropa[3α,5]-5α-pregnane (AMDCP)

(20*S*)-22-Hydroxymethyl-6β-methoxy-3α,5-dihydro-3′H-cyclopropa[3α,5]-5α-pregnane [16] (250 mg) was dissolved in pyridine (2 mL) and acetic anhydride (2 mL). The solution was heated at 80°C for 1 h. The solvent was evaporated to isolate the crude product (280 mg), which was then purified by recrystallization from methanol (140 mg) to yield AMDCP (m.p. 122–123°C, mass spectrum: M^+^ 388). Anal. calcd for C_25_H_40_O_3_, C 77.27, H 10.38% (found: C 77.06, H 10.44%) for the X-ray structure [17]. AMDCP was administered orally to rats at doses of 1, 5, 10, 15 or 20 mg/kg body weight (5 mL/kg body weight).

### Acute toxicity test and experimental animals

Healthy male and female ICR mice (6–7 weeks old) were obtained from the Animal House, Faculty of Medicine, University of Malaya, Kuala Lumpur (Ethic No. PM/27/07/2010/MAA (R)). The mice weighed between 25 and 30 g. The animals were fed a standard rat pellet diet and tap water. The acute toxicity study was used to determine a safe dose for AMDCP. Thirty-six mice (18 males and 18 females) were randomly assigned into 3 groups: vehicle (10% Tween 20, 5 mL/kg), low-dose (100 mg/kg) and high-dose (2000 mg/kg) of AMDCP (10% Tween 20, 5 mL/kg) according to OECD [18]. Prior to dosing, the animals were fasted overnight (i.e., receiving water but not food). Food was withheld for an additional 3 to 4 h after dosing. The animals were observed continuously for 30 min, they were then monitored frequently (2, 4, 8, 24 and 48 h) for the onset of any clinical or toxicological symptoms. Mortality, if any, was observed over a period of 2 weeks. The animals were sacrificed on the 15^th^ day. Histological, hematological and serum biochemical parameters were determined according to the OECD [18]. The study was approved by the Ethics Committee for Animal Experimentation, Faculty of Medicine, University of Malaya, Malaysia. During the experiments, all animals received humane care according to the criteria outlined in the “Guide for the Care and Use of Laboratory Animals” prepared by the National Academy of Sciences and published by the National Institutes of Health.

RETRACTED

### Experimental animals for gastric mucosal lesions

Healthy adult *Sprague Dawley* male rats were obtained from the Experimental Animal House, Faculty of Medicine. The rats were divided randomly into 8 groups of 6 rats each. Each rat that weighed between 180 and 220 g was placed individually in a separate cage (1 rat per cage) with wide-mesh wire bottoms to prevent coprophagia during the experiment. The animals were maintained on a standard pellet diet and tap water. The study was approved by the Ethics Committee for Animal Experimentation, Faculty of Medicine, University of Malaya, Malaysia.

### Gastric mucosal lesion-induction by ethanol

The rats were fasted for 24 h, but they had access to drinking water up to 2 h prior to the experiment. The negative control group (group 1) was orally administered 10% Tween 20 (5 mL/kg). The ethanol control group (group 2) was orally administered 10% Tween 20 (5 mL/kg). The reference control group (group 3) received a single oral dose of 20 mg/kg omeprazole (10% Tween 20, 5 mL/kg). AMDCP at doses of 1, 5, 10, 15 and 20 mg/kg (10% Tween 20, 5 mL/kg) was orally administered to the experimental groups (groups 4–8). One hour after treatment, 10% Tween 20 (5 mL/kg) was orally administered to the negative control group, and absolute ethanol was orally administered to the rest of the groups to induce gastric mucosal lesions (5 mL/kg). The rats were euthanized 1 h later with an overdose of xylazine and ketamine anesthesia, and their stomachs were immediately excised.

### Measurement of gastric juice acid content (pH)

Samples of gastric contents were analyzed for hydrogen ion concentration by pH metric titration with 0.1 N NaOH solutions using a digital pH meter.

### Determination of gastric wall mucus (GWM)

The gastric wall mucus was evaluated according to the modified procedure of Corne *et al.* [19]. Glandular stomach segments were separated from the lumen, weighed and transferred immediately to 10 mL of a 0.1% w/v Alcian blue solution (in a 0.16 M sucrose solution buffered with 0.5 mL of sodium acetate, pH 5). The tissue was stained for 2 h in Alcian blue. Excess dye was removed by 2 consecutive rinses with 10 mL of 0.25 M sucrose. The dye that complexed with the gastric wall mucus was extracted using 10 mL of 0.5 M magnesium chloride. This mixture was intermittently shaken for 1 min at 30 min intervals over 2 h. Four milliliters of the blue extract was then vigorously shaken with an equal volume of diethyl ether. The resulting emulsion was centrifuged at relative centrifugal force (RCF)  = 2361× g for 10 min. The absorbance of the aqueous layer was recorded at 580 nm. The quantity of Alcian blue that was extracted from the wet glandular tissue was then calculated.

RETRACTED

### Macroscopic gastric lesions evaluation

The presence of elongated bands of red hemorrhagic lesions parallel to the long axis of the stomach is a symptom of mucosal lesions of the gastric mucosa. The gastric mucosa of each rat was then examined for damage. The length and width of the lesion (mm) were measured using a planimeter (10×10 mm^2^  =  lesion area) under a dissecting microscope (1.8×). The ulcerated area was measured by counting the number of small squares (2 mm ×2 mm) covering the length and width of each mucosal lesion band. The sum of the areas of the all lesions for each stomach was used to calculate the mucosal lesion area (LA), in which sum of the small squares ×4×1.8 =  LA (mm^2^), according to the previously used protocol [20]. The inhibition percentage (I%) was calculated using the following formula according to the method of Abdulla *et al.* [21].


### Histological evaluation of gastric lesions

Specimens from the gastric walls of each rat were fixed in 10% buffered formalin and processed in a paraffin tissue processing machine. Sections of the stomach were sliced at a thickness of 5 µm and stained with hematoxylin and eosin for histological evaluation [13], [21].

### Immunohistochemistry

Tissue section slides were heated at 60°C for approximately 25 min in a hot air oven (Venticell, MMM, Einrichtungen, Germany). The tissue sections were de-paraffinized in xylene and rehydrated using an alcohol gradient. The antigen retrieval process was performed in 10 mM sodium citrate buffer. Immunohistochemical staining was conducted according to the manufacturer's protocol (Dako Cytomation, USA). Briefly, endogenous peroxidase was blocked in a peroxidase blocking solution (0.03% hydrogen peroxide containing sodium azide) for 5 min. Tissue sections were washed gently with washing buffer and subsequently incubated with Hsp70 (1∶500) or Bax (1∶200) biotinylated primary antibodies for 15 min. The sections were rinsed gently with washing buffer and placed in a buffer bath. The slides were then placed in a humidified chamber with a sufficient amount of streptavidin – HRP (streptavidin conjugated to horseradish peroxidase in phosphate-buffered saline (PBS) containing an anti-microbial agent). The slides were incubated for 15 min. Subsequently, the tissue sections were rinsed gently in washing buffer and placed in a buffer bath. A diaminobenzidine-substrate-chromogen was added to the tissue sections and incubated for 5 min, followed by washing and counterstaining with hematoxylin for 5 sec. The sections were then dipped in weak ammonia (0.037 M/L) 10 times, rinsed with distilled water and cover slipped. Positive immunohistochemical staining was observed as brown stains under a light microscope.

RETRACTED

### Biological activity of gastric homogenate

#### Sample preparations

The gastric tissue homogenate from each rat was prepared for PGE_2_ and MDA assays. The entire experiment was performed at 4°C. Gastric tissue was cut into 3 small pieces (approximately 200 mg for each), and the exact weight of each piece was recorded [22]. The tissues were homogenized in a teflon homogenizer (Polytron, Heidolph RZR 1, Germany) using the appropriate buffer. The amount of buffer used was dependent on the weight of the tissue used. After centrifugation at 4,500 rpm for 15 min at 4°C, the supernatant was used for the PGE_2_ and MDA assays.

#### Measurement of membrane lipid peroxidation (MDA)

The rate of lipoperoxidation in the gastric mucosal membrane was determined by measuring the level of MDA using the Thiobarbituric Acid Reactive Substances test. The tissues were washed with phosphate-buffered saline to minimize the interference of hemoglobin and to remove blood adhered to the gastric mucosa. The stomachs were homogenized with 10% of the tissue using potassium phosphate buffer. Then, 250 μL of homogenate were incubated at 37°C for 1 h, 400 μL of 35% perchloric acid was added, and the mixture was centrifuged at 4,500 rpm for 20 min at 4°C. The supernatant was removed, mixed with 400 μL of 0.6% thiobarbituric acid and incubated at 95–100°C for 1 h. After the homogenate was cooled, the absorbance was measured at 532 nm. A standard curve was generated using 1,1,3,3-tetramethoxypropane. The results were expressed as nM of MDA/mg of protein. The concentration of the protein was measured using the method described by Bradford [23], which is based on the interaction of Coomassie Blue G250 dye with proteins. The amount of total protein in each tissue sample was measured after the lesions were induced by ethanol treatment. The interaction between the high molecular weight proteins and the dye causes a shift in the dye to its anionic form, which exhibits a strong absorbance at 595 nm. Solutions of albumin standard, distilled water, buffer (Borate 50 mM, Tris 25 mM, HEPES 100 mM and Phosphate 100 mM) and each sample were added to the wells. For sample preparation, 2 μL of sample and 38 μL of buffer were added to each well. Then, 200 μL of Bradford's solution (diluted 5×) was added to each well. After a 5 min incubation, absorbance at the wavelength of 595 nm was recorded, according to the Bradford method [23].

RETRACTED

#### Measurement of PGE_2_ formation using enzyme immunoassays

The gastric mucosa was weighed, minced with scissors, and homogenized at 4°C in PBS buffer. Homogenates were centrifuged at 1400 rpm for 10 min. The supernatants were analyzed by PGE_2_ assay using a PGE_2_ Monoclonal Enzyme Immunoassay Kit (Sigma-Aldrich, Malaysia).

#### Measurement of protein concentration

Protein concentrations (mg/mL tissue) were determined using the Biuret reaction, as described by Gornall *et al.* [24].

### Statistical analysis

All values are reported as the means ± S.E.M. The statistical significance of the differences between groups was assessed using a one-way ANOVA. A p-value of *p<0.05* was considered to be significant.

## Results

### Acute toxicity study

An acute toxicity study did not show any sign of toxicity in any groups within 14 days. There were no histological signs of hepatic or renal toxicity. Moreover, the blood biochemistry analysis appeared normal.

### Effect of AMDCP on mucosal lesion area

The experimental groups showed significant prevention of gastric lesion formation as well as a significant increase in the percent inhibition of gastric mucosal lesions (Figure 1).

**Figure 1:** Effect of AMDCP on gastric mucosal lesions and inhibition percentage in rats. Inhibition of gastric lesions (%) is indicated in brackets above the columns. Groups 2 and 3 represent the ethanol control group and the reference control group, respectively. The experimental groups are presented as groups 4–8. All values are expressed as the means ± standard error of the mean. Mean difference is significant at the *p*<0.05 level (one-way between groups ANOVA with post-hoc analysis). * significant when compared with the group 2. # significant when compared with the group 3.

### Macroscopic evaluation of gastric lesions

The gastroprotective activity of AMDCP in the ethanol-induced gastric lesion model is shown in Figure 2. The results showed that rats in the reference control group and in the experimental groups showed a pronounced reduction in the formation of gastric mucosal lesions compared with the ethanol control group (Figure 2). Ethanol produced extensive visible red hemorrhagic lesions of the gastric mucosa. AMDCP dramatically suppressed the formation of mucosal lesions and produced a notable flattening of the gastric mucosal folds in rats pre-treated with 20 mg/kg of AMDCP (Figure 2). The remarkable inhibition of gastric mucosal lesions in rats pre-treated with 10 mg/kg of AMDCP (group 7) was comparable with the reference control group (omeprazole, 20 mg/kg) (Figure 2).

RETRACTED

**Figure 2:** Macroscopic appearance of the gastric mucosa in rats. The negative control group showed no injuries to the gastric mucosa (A). Severe injuries were observed in the gastric mucosa of the ethanol control group. Ethanol treatment produced extensive visible hemorrhagic lesion of the gastric mucosa (B). The reference control group, treated with omeprazole (20 mg/kg), showed milder injuries to the gastric mucosa compared to the injuries observed in the ethanol control group (C). Group 4 (1 mg/kg AMDCP) showed moderate injuries to the gastric mucosa (D). Group 5 (5 mg/kg AMDCP), mild injuries were observed in the gastric mucosa. AMDCP reduced the formation of gastric lesions induced by ethanol (E). Groups 6, 7, and 8 (10, 15, and 20 mg/kg AMDCP, respectively) showed no injuries to the gastric mucosa. Instead, flattening of the gastric mucosa was observed (F, G and H).

### Gastric mucosal wall evaluation

Treatment with ethanol caused a significant decrease in the mucus content of the gastric wall in the ethanol control group (Figure 3). The depleted gastric mucus was significantly replenished in the experimental groups. It was also found that the experimental groups significantly increased the amount of gastric mucus (Figure 3).

**Figure 3:** Effect of AMDCP on ethanol-induced changes in the Alcian blue binding capacity of gastric mucosa, gastric mucosal lesions area and inhibition percentage in the gastric mucosa of rats. Groups 1, 2 and 3 represent the negative control group, the ethanol control group and the reference control group, respectively. The experimental groups are presented as groups 4–8. All values are expressed as the means ± standard error of the mean. Mean difference is significant at the *p*<0.05 level (one-way between groups ANOVA with post-hoc analysis). * significant when compared with the group 2. # significant when compared with the group 3.

### pH of gastric content

The acidity of the gastric content in the experimental groups was decreased significantly compared with that of the ethanol control group (*p*<0.05) (Figure 4).

**Figure 4:** Effect of AMDCP on the pH of gastric content. Groups 1, 2, and 3 represent the negative control group, the ethanol control group and the reference control group, respectively. The experimental groups are presented as groups 4–8. All values are expressed as the means ± standard error of the mean. Mean difference is significant at the *p*<0.05 level (one-way between groups ANOVA with post-hoc analysis). * significant when compared with the group 2. # significant when compared with the group 3.

RETRACTED

### Histological evaluation of gastric lesions

Histological evaluation of the ethanol-induced gastric lesions in the ethanol control group showed extensive damage to the gastric mucosa, necrotic lesions penetrating deeply into the mucosa, extensive edema and leukocyte infiltration of the submucosal layer (Figure 5). Rats in the experimental groups had better protection of the gastric mucosa compared with the controls as observed by a reduction of mucosal lesions, submucosal edema and leukocyte infiltration (Figure 5). AMDCP has been shown to exert protective effects in a dose-dependent manner.

**Figure 5:** Histological study of ethanol-induced gastric mucosal damage in rats. In the negative control group no injuries to the gastric mucosa were observed (A). The ethanol control group showed severe disruption to the surface epithelium (black arrow), gastric lesions penetrating deeply into the mucosa, and extensive edema of the submucosal layer (yellow arrow), and leukocyte infiltration (blue arrow) was present (B). The reference control group showed mild disruption of the surface epithelium mucosa. There was edema and leukocyte infiltration of the submucosal layer (C). Group 4 (1 mg/kg AMDCP) exhibited moderate disruption of the surface epithelium. There was edema with leukocyte infiltration of the submucosal layer (D). Group 5 (5 mg/kg AMDCP) had mild disruption of the surface epithelium. There was no edema or leukocyte infiltration of the submucosal layer (E). Groups 6, 7 and 8 (10, 15 and 20 mg/kg AMDCP, respectively) did not show any disruption to the surface epithelium. There was no edema or leukocyte infiltration of the submucosal layer (F, G and H) (H & E stain, 10x).

### Immunohistochemistry

The immunohistochemical results of the experimental groups demonstrated that the pre-treatment caused over-expression of Hsp70 protein. The expression of Hsp70 protein in the experimental groups was up-regulated compared to Hsp70 expression in the control groups (Figure 6). Immunohistochemical staining of Bax protein demonstrated that the experimental groups showed decreased expression of the Bax protein. Expression of Bax protein in the experimental groups was down-regulated compared to the ethanol control group (Figure 6).

**Figure 6:** Immunohistochemical analysis of Hsp70 and Bax proteins expression in the stomachs of rats with ethanol-induced gastric mucosal lesions. Immunohistochemical staining of the Hsp70 proteins (First row) and Bax proteins (second row); the negative control group (A and D), the ethanol control group (B and E) and the treated group with 20 mg/kg AMDCP (C and F). Arrows indicate the proteins *in situ* (10x).

RETRACTED

### PGE_2_, MDA levels and protein concentration of the gastric tissue homogenate

In gastric tissue homogenates, PGE_2_ activity in the ethanol control group was significantly lower than that in the negative control group (Figure 7). Administration of AMDCP before ethanol treatment significantly increased the level of PGE_2_ compared to that of the ethanol control group. Administration of ethanol significantly increased the level of MDA in gastric homogenate in the ethanol control group compared to the negative control group. Administration of AMDCP decreased the MDA level in gastric tissues compared to the ethanol control group (Figure 8). Protein concentration in gastric homogenates was significantly decreased in the ethanol control group compared with the negative control group. Administration of AMDCP significantly increased the protein content of gastric homogenate compared with the ethanol control group (Figure 9).

**Figure 7:** Effects of AMDCP on PGE2 in the gastric mucosal homogenates from rats. Groups 1, 2 and 3 represent the negative control group, the ethanol control group and the reference control group, respectively. The experimental groups are presented as groups 4–8. All values are expressed as the means ± standard error of the mean. Mean difference is significant at the *p*<0.05 level (one-way between groups ANOVA with post-hoc analysis). * significant when compared with the group 2. # significant when compared with the group 3.

**Figure 8:** Effect of AMDCP on the level of MDA in the gastric mucosal homogenates from rats. Groups 1, 2 and 3 represent the negative control group, the ethanol control group and the reference control group, respectively. The experimental groups are presented as groups 4–8. All values are expressed as the means ± standard error of the mean. Mean difference is significant at the *p*<0.05 level (one-way between groups ANOVA with post-hoc analysis). * significant when compared with the group 2. # significant when compared with the group 3.

**Figure 9:** Effect of AMDCP on protein concentration in the gastric mucosal homogenates from rats. Groups 1, 2 and 3 represent the negative control group, the ethanol control group and the reference control group, respectively. The experimental groups are presented as groups 4–8. All values are expressed as the means ± standard error of the mean. Mean difference is significant at the *p*<0.05 level (one-way between groups ANOVA with post-hoc analysis). * significant when compared with the group 2. # significant when compared with the group 3.

## Discussion

Imbalance between the protective and aggressive mechanisms of the mucosa, which may be triggered by several endogenous factors and aggressive exogenous factors, is the main cause of peptic ulcers [25]. Ethanol treatment produces necrotic lesions by direct necrotizing action, which in turn reduces defensive factors, such as the secretion of bicarbonate and the production of mucus [26]. Ethanol can reach the mucosa by disrupting the mucus-bicarbonate barrier, causing cell rupture in the walls of blood vessels. These effects are most likely due to biological actions, such as lipid peroxidation, formation of free radicals, intracellular oxidative stress, changes in permeability and depolarization of the mitochondrial membrane prior to cell death [27]. In addition, ethanol treatment produces linear hemorrhagic lesions, extensive submucosal edema, mucosal friability, inflammatory cell infiltration, and epithelial cell loss in the stomach. These symptoms are typical characteristics of alcohol injury [28].

RETRACTED

In the present study, AMDCP did not show any signs of toxicity or mortality in any of the acute toxicity tests performed. Behavioral changes, such as irritation, restlessness, respiratory distress, abnormal locomotion and catalapsy, over a period of 14 days were not observed. The observed decrease in acidity and increase in the gastric wall mucus in response to AMDCP is consistent with the results reported previously by Al-Attar [29]. Similarly, Hajrezaie *et al.* [10] reported a reduction in gastric acidity in treated animals. Omeprazole exhibits both an anti-secretory and a protective effect [30]. Omeprazole, a proton pump inhibitor (PPI), offered some protection to the gastric mucosa and has been widely used as an acid inhibitor in the treatment of disorders related to gastric acid secretion [31]. In addition to its anti-secretory effect and effectiveness in acid-dependent ulcer models, omeprazole is also effective in acid independent models, such as in the ethanol-ulcer model. In the ethanol-ulcer model, omeprazole exhibits mucosal protection at doses that do not inhibit secretion [32], [33]. Similarly, H2 blocking drugs can also induce gastroprotection at non-anti-secretory doses [34].

Absolute alcohol extensively damaged the gastric mucosa, leading to increased neutrophil infiltration into the gastric mucosa. Activation and infiltration of neutrophils appear to be involved in the initial processes of lesion formation. In the present study, histopathology results also revealed the protection of gastric mucosa and inhibition of leukocyte infiltration into the gastric wall of rats pre-treated with AMDCP. Previous studies demonstrated that the reduction of neutrophil infiltration into gastric lesion promotes the prevention of gastric mucosal lesions in rats [10], [21], [35]. Wasman *et al.* [36] showed that oral administration of the *Polygonum minus* aqueous leaf extract prior to ethanol administration significantly decreased neutrophil infiltration into the gastric mucosa. In the present study, we observed flattening of the mucosal folds, which suggests AMDCP exerts a gastroprotective effect. Relaxation of circular muscles may protect the gastric mucosa by flattening the folds. Flattening of the mucosal folds increases the mucosal area exposed to necrotizing agents and reduces the volume of the gastric irritants on the rugal crest [21], [36]. It was shown that enhanced gastric motility may contribute to the development of gastric mucosal lesions [6]. Ethanol produces a marked contraction of the circular muscles of the rat fundic strip. Such a contraction can lead to mucosal compression at the site of the greatest mechanical stress, the crests of mucosal folds, leading to necrosis and lesion [20]. Gastric tissue homogenates from experimental groups showed significantly decreased levels of MDA and elevated levels of PGE_2_ in response to oxidative stress due to absolute ethanol administration. MDA is the final product of lipid peroxidation and is used to determine the level of lipid peroxidation in tissues [37]. PGE_2_ plays an important role in the regulation of gastric mucus secretion [38]. PGE_2_ has exhibited protective effects in various models of gastric lesion [39], [40]. PGE2, the most abundant gastrointestinal prostaglandin, regulates functions of the gut, including motility and secretion. PGE2 has also been shown to protect the stomach by the activating EP receptors [41] and by modulating gastrointestinal mucosal integrity [5]. The results of the present study suggest that the gastroprotective effect of AMDCP is partially mediated by PGE_2_. A direct measurement of the PGE_2_ mucosal level confirmed that its biosynthesis was significantly enhanced by AMDCP. It has been shown that prostaglandins influence virtually every component of the mucosal defense [38]; stimulating mucus and bicarbonate secretion, maintaining mucosal blood flow, enhancing the resistance of epithelial cells to injury induced by cytotoxins and inhibiting leukocyte recruitment [42].

RETRACTED

Hsp70 proteins defend cells from oxidative stress or heat shock. Ethanol-generated ROS normally inhibits the expression of Hsp70 and increases the expression of Bax. Hsp70 prevents partially denatured proteins from aggregating and allows them to refold. The over-expression of Hsp70 observed in this study suggests that AMDCP protected the gastric tissues by up-regulating Hsp70.

## Conclusion

In conclusion, the acute toxicity study demonstrated that rats treated with AMDCP (2000 mg/kg) manifested no abnormal signs. This synthetic steroid could significantly protect the gastric mucosa against ethanol-induced injury. This protection was ascertained grossly by a significant increase in the gastric wall mucus in comparison with the ethanol control group. Additionally, a reduction of mucosal lesions in the gastric wall and reduction or inhibition of edema and leukocyte infiltration in the submucosal layers was shown histologically. Immunohistochemical staining for the Hsp70 and Bax proteins showed over-expression of the Hsp70 protein and down-regulation of the Bax protein in rats pre-treated with the synthetic steroid. Assays for the levels of PGE_2_ and MDA in gastric tissue homogenates revealed that AMDCP significantly increased the amount of PGE_2_ and decreased the level of lipid peroxidation (MDA) in the experimental groups compared to the ethanol control group. This study provides evidence that AMDCP possesses a gastroprotective effect, which is partially due to the preservation of gastric mucus secretion, increased production of Hsp70 protein, and the presence of antioxidant enzymes.
